RETRACTED

# Exosomes function as nanoparticles to transfer miR-199a-3p to reverse chemoresistance to cisplatin in hepatocellular carcinoma

**DOI:** 10.1042/BSR20194026

**Published:** 2020-06-06

**Authors:** Kun Zhang, Chu-xiao Shao, Jin-de Zhu, Xin-liang Lv, Chao-yong Tu, Chuan Jiang, Min-jie Shang

**Affiliations:** 1 Department of Hepatobiliary Surgery, Lishui Municipal Central Hospital, Zhejiang, China; 2 Department of Hepatobiliary and Pancreas Minimally Invasive Surgery, Zhejiang Provincial People’s Hospital, Zhejiang, China

**Keywords:** DDP, Exosome, hepatocellular carcinoma, Huh-7/DDP, miR-199a-3p

## Abstract

Hepatocellular carcinoma (HCC) is a frequently seen malignant tumor globally. The occurrence of cisplatin (DDP) resistance is one of the main reasons for the high mortality of HCC patients. Therefore, it is of great theoretical significance and application value to explore the mechanism of chemotherapy resistance. Drug resistance can be modulated by exosomes containing mRNAs, micro RNAs (miRNAs) and other non-coding RNA (ncRNAs). Exosomal miR-199a-3p (Exo-miR-199a-3p) was subjected to extraction and verification. Whether exo-miR-199a-3p could make HCC cells sensitive to DDP *in vitro* was verified via flow cytometry, Cell Counting Kit-8 (CCK-8) assay, immunofluorescence assay and Transwell assay. Intravenous injection of exo-miR-199a-3p and intraperitoneal injection of DDP were carried out *in vivo*. Moreover, the possible targets of miR-199a-3p were screened through bioinformatics analysis, which were ascertained by Western blotting (WB). Then, miR-199a-3p levels in human normal liver epithelial cell line HL-7702 and HCC cell lines HuH7 and HuH7/DDP were elevated in a concentration-dependent manner. Exo-miR-199a-3p has abilities to adjust underlying targets and conjugate cells, to repress cells to invade, stimulate their apoptosis and abate their ability. Additionally, the caudal injection of exo-miR-199a-3p reversed the chemoresistance of tumors and slowed down their growth in the body owing to the up-regulation of miR-199a-3p and down-regulation of underlying target proteins in tumors. Finally, exo-miR-199a-3p was found to overturn the HCC’s resistance to DDP, and it may function in DDP-refractory HCC therapy as an underlying option in the future.

## Introduction

Hepatocellular carcinoma (HCC), which is one of the most common malignancies all over the world, is a major cause of death associated with cancer [1]. The global death of HCC has been recorded 700,000 annually [2]. The growth of HCC can be facilitated by chemicals, viruses and congenital or acquired metabolic diseases [3,4]. Although a large variety of therapies have been used for treating liver cancer, the prognosis of HCC is still poor, and its 5-year survival rate is below 20% due to its high metastasis and recurrence rates [5,6]. Hence, it is important to work out the possible therapeutic targets of HCC. Besides, the drug resistance to DDP, a first-line chemotherapeutic drug for clinical treatment of HCC, seriously affects its efficacy and is one of the main reasons for the low 5-year survival rate of clinical patients. Therefore, it is necessary to find alternative targets of drug resistance to reduce the occurrence of drug resistance [7]. Currently, there is still no effective prediction and treatment for the development of HCC chemoresistance [8]. Therefore, it is of great theoretical significance and application value to study the mechanism of HCC chemoresistance [9]. Studies have found the diverse mechanism of DDP resistance, including drug-related molecular and genetic changes [10], drug uptake accumulation and transport disorders [11] and DNA repair enhancement or increased tolerance of DNA damage [12]. In addition, more and more studies have proved that miRNAs and exosomes are involved in drug resistance in recent years [13,14].

RETRACTED

MiRNAs are a kind of endogenous non-coding small RNAs of approximately 19–24 nucleotides in length, which are mainly found in eukaryotes [15]. miRNA regulates the pathophysiological processes of various diseases through linking to target mRNA 3′UTR by base-complementary pairing to inhibit mRNA translation or degradation [16]. Besides, numerous studies have found that miRNAs play crucial parts in tumorigenesis, metastasis and drug resistance [17,18]. In HCC, miRNA is not only an effective biomarker [19], but also has an effect of regulating HCC cell proliferation, apoptosis and chemotherapeutic drug sensitivity [20]. MiR-199a-3p, a non-coding RNA, inhibits the occurrence and development of tumors such as prostate cancer [21], esophageal cancer [22] and clear cell renal cell carcinoma [23] by modulating cells to proliferate, invade and migrate. More importantly, miR-199a-3p has been revealed to enhance the sensitivity of cholangiocarcinoma cells [24], breast cancer cells [25] and ovarian cancer cells [26] to chemotherapeutic drugs. Therefore, the sensitivity to chemotherapy can be strengthened through up-regulating miR-199a-3p expression in the tumor microenvironment and cells. In HCC, miRNA-199a-3p has also been identified as an important biomarker [27] and can inhibit tumorigenesis and progression by regulating related target genes [28,29]. However, whether miR-199a-3p can enhance the HCC cell’s sensitivity to DDP has not been reported.

An exosome is a nano-sized vesicle body that is actively secreted by cells with a diameter of 30–150 nm and a lipid bilayer structure with an uniform size [30]. As a vesicle structure that transmits signals between cells, exosomes remarkably function in tumor proliferation [31], invasion [32] and drug resistance [33]. Besides, research has found that exosomes are able to regulate the resistance of tumor cells by transferring proteins, DNAs, RNAs and other molecules [14]. For example, in gastric cancer, exosomal transfer of tumor-correlated miR-21 originated from macrophages can cause HCC cell’s resistance to DDP [34]. It has been manifested in research that exosomal miRNAs exert a pivotal effect in the pathogenesis of HCC [35,36], but whether exosomal miRNA can affect HCC cell resistance is still rarely reported.

RETRACTED

In the present research, emphasis was put on DDP-refractory HCC, and the chemoresistance to DDP was overturned via systemic injection of exosomes containing miR-199a-3p mimics. In the first place, miR-199a-3p mimics were injected into HCC cells in a direct manner to ascertain that miR-199a-3p is capable of modulating the sensitivity of DDP treatment. Thereafter, exosomal miR-199a-3p was extracted, and then a train of assays were implemented to ascertain that these nanoparticles had the ability to overturn the drug resistance inside and outside the body. Bioinformatics prediction was adopted for the screening of possible target genes of miR-199a-3p in cancer cells, which was then demonstrated by WB. The research results imply that miR-199a-3p may be a treatment target for DDP-refractory HCC patients in further research.

## Materials and methods

### Cell culture

The Cell Bank of the Chinese Academy of Sciences (Shanghai, China) provided the human immortalized liver epithelial cell line HL-7702, the human embryo kidney epithelial cell line HEK293T, and the human HCC cell line Huh-7, and Oulu Biotechnology (Shanghai, China) provided the human DDP-resistant HCC cell line Huh-7/DDP, with the largest bearable dose of DDP of 800 ng/ml according to the guidelines. DMEM acquired from Gibco (China) with 10% fetal bovine serum (FBS) from the same company and 1% penicillin/streptomycin provided by Beyotime Biotechnology (Nantong, China) were utilized for cell culture in a moist incubator with 5% CO_2_ at 37°C.

### Transfection of cells

HL-7702, Huh-7 and Huh-7/DDP Cells (3 × 10^5^) were seeded into six-well plates for cell transfection upon cell fusion of 40–60%. By reference to the guidance of the manufacturer, Opti-MEM and Lipofectamine 2000 were employed to treat different cells following inoculation in varying plates. Tube A was made of 5 μl/well of lipofectamine 2000 (Thermo, U.S.A.) and 250 μl of Opti-MEM culture medium (Gibco, U.S.A.). Tube B was made of miR-199a-3p mimics and negative control (RiboBio, China) (5 μl/well) in 250 μl of Opti-MEM culture medium. The working concentration of miR-199a-3p mimics was 50 nM. Tube A was incubated at room temperature for 5 min before mixed with tube B for 20 min. After that, PBS was utilized for cell rinsing, and following 5 h of transfection, complete medium was use to replace the original medium.

RETRACTED

### Cell viability experiment

Cell Counting Kit-8(CCK-8) (MYBiotech, China) experiment for cell viability was implemented. Huh-7 or Huh-7/DDP cells received inoculation into a 96-well plate and treatment or incubation with exosomes, followed by 48 h of exposure to different doses of DDP (Jiangsu Haosen, China). Following transfection, plate wells were added with CCK-8 solution (10 μl), and cells in these wells underwent 1 h of incubation at 37°C. Thereafter, cell viability was determined by detecting the optical density (OD) at 450 nm using a microplate reader (Thermo). This experiment was implemented thrice at least, and the cell viability was worked out referring to formula:

$$\text{Inhibition ratio}=\frac{\left(\text{control group OD - experimental group OD}\right)}{\left(\text{control group OD - blank group OD}\right)}\times 100\%$$

### Cell invasion experiment

Cell invasion capacity was assessed via Transwell assay. The cells were raised with varying exosomes for 24 h, about 1 × 10^5^ cells of which were placed in the upper chamber containing serum-free medium (200 μl), whereas the lower chamber was added with 10% FBS-supplemented complete medium (600 μl) for chemotaxis. Then, cells invaded the membrane coated with Matrigel. Finally, the cells undergoing invasion were dyed and quantified under a light microscope, and Transwell assay was carried out thrice.

### Isolation of exosomes

In the first place, the culture medium of HEK293T cells was obtained, and then centrifuged at 300 × ***g*** and 3000 × ***g*** to remove debris and cells, respectively. Subsequent to supernatant centrifugation at 10000 × ***g*** for 30 min, larger sloughy vesicles were thrown away. In the end, the supernatant centrifugation was carried out at 110,000 × ***g*** for 70 min, and the pellet containing exosomes was subjected to resuspension in 1× PBS and filtering using filters (0.2 μm). Considering the exosomes enriched with miR-199a-3p, cells transfected with miR-199a-3p mimics were incubated with the conditioned medium (CM) for 48 h. After that CM was collected and used to extract exosomes from the medium, following previously described standard procedures [37]. The assay was implemented at 4°C, and exosomes in plasma were extracted by reference to the guideline of the Total Exosome Isolation kit acquired from Invitrogen. The concentration of exosomes, purified from cell culture supernatants or plasma were determined using NanoSight NS300 (Malvern Instruments) [38].

RETRACTED

### Transmission electron microscopy

Glutaraldehyde (2.5%) in PBS (pH 7.2) was dropwise injected into exosomes overnight at 4°C during transmission electron microscopy. Following PBS rinsing, 1% osmium tetroxide was utilized for immobilizing specimens at room temperature for 1 h. After that, these specimens underwent embedding in gelatin (10%), immobilization in glutaraldehyde at 4°C and slicing into sections with the volume of <1 mm^3^. Thereafter, the specimens were subjected to dehydration with alcohol at gradient concentrations (30%, 50%, 70%, 90%, 95% and 100%), and propylene oxide was added to replace pure alcohol and mixed with Quetol-812 epoxy resin at gradient concentrations (25%, 50%, 75% and 100%) to permeate the specimens. Following embedding in pure Quetol-812 epoxy resin, all specimens were aggregated at 35°C for 12 h, at 45°C for 12 h, and at 60°C for 24 h. Subsequent to observation using a FEI Tecnai T20 transmission electron microscope at 120 kV, a Leica UC6 ultramicrotome was employed to cut 100 nm ultrathin sections, and the sections were dyed by uranyl acetate for 10 min and by lead citrate for 5 min at indoor temperature.

### PKH67 dying

Lipid bilayer marking was implemented using PKH67 Fluorescent Cell Linker Kits acquired from Sigma. First, Diluent C was utilized to re-suspend exosomes, and 0.4 ml of PKH67 ethanol staining solution was added to 100 μl Diluent C to prepare a 4 × 10^−6^ M staining solution. Then, 100 μl exosome suspension liquid was pipetted to mix with 100 μl staining solution. Subsequently, the cell/staining suspension was incubated for 5 min, and after periodic mixing, 200 μl of serum was added to terminate the dying through incubation for 1 min. Afterwards, the dyed exosomes underwent 1× PBS rinsing and resuspension in new sterile conical polypropylene tubes. Finally, the cell culture medium was added with an appropriate quantity of dyed exosomes for four hours of incubation, followed by photographing.

### Extraction of proteins and WB

The newly added protease inhibitor and the lysis buffer (SDS) were applied for protein separation. Subsequent to separation through SDS-PAGE, the lysates were transferred onto a polyvinylidene fluoride membrane acquired from Roche. Then the membrane was blocked with 2% BSA, followed by incubation with anti-CD63 and anti-TSG 101 from Santa Cruz, and anti-Alix, ZEB1 antibody, MTOR antibody, DNMT3A antibody and GAPDH antibody from Abcam at 4°C overnight. Then the membrane underwent incubation with the proper secondary antibodies, and the protein expression in cells was measured with GAPDH as an internal reference.

RETRACTED

### RNA extraction and qRT-PCR

TRIzol reagent (Beyotime Biotechnology, Nantong, China) was employed to extract exosomal RNA and total cellular RNA. The experimental procedure was carried out in strict accordance with the kit instructions. RT of RNA into cDNA was implemented with the use of reverse transcriptase provided by TaKaRa (Dalian, China). The two-step PCR amplification standard procedure was performed on the machine. After the amplification, the cycle threshold number (Ct value) was obtained. Then two replicate wells were set for each sample, and the gene expression level was calculated by 2^−ΔΔCt^ method, where ΔΔCt = experimental group ΔCt (target gene Ct − internal reference gene Ct) − control group ΔCt (target gene Ct − internal reference gene Ct). Sequences of primers for miRNA related sequence were showed in Table 1.

**Table 1:** Sequences of primers for qRT-PCR and miRNA related sequence

Name		Sequence
MTOR	Forward	5′- ATGCTTGGAACCGGACCTG -3′
	Reverse	5′- TCTTGACTCATCTCTCGGAGTT -3′
ZEB1	Forward	5′- GCCAATAAGCAAACGATTCTG -3′
	Reverse	5′- TTTGGCTGGATCACTTTCAAG -3′
GAPDH	Forward	5′- GATCATCAGCAATGCCTCC -3′
	Reverse	5′- TCCACGATACCAAAGTTGTC -3′
U6	Forward	5′- CTCGCTTCGGCAGCACA -3′
	Reverse	5′- AACGCTTCACGAATTTGCGT -3′
miR-199a-3p	Forward	5′- ACACTCCAGCTGGGACAGTAGTCTGCACAT -3′
	Reverse	5′- CTCAACTGGTGTCGTGGAGTCGGCAATTCAGTTGAGTAACCAAT-3′
DNMT3A	Forward	5′- CCGATGCTGGGGACAAGAAT -3′
	Reverse	5′- CCCGTCATCCACCAAGACAC -3′
Alix	Forward	5′- ATGGCGACATTCATCTCGGTG-3′
	Reverse	5′- CGCTTGGGTAAGTCTGCTGG -3′
CD63	Forward	5′- CAGTGGTCATCATCGCAGTG -3′
	Reverse	5′- ATCGAAGCAGTGTGGTTGTTT -3′
TSG101	Forward	5′- GAGAGCCAGCTCAAGAAAATGG -3′
	Reverse	5′- TGAGGTTCATTAGTTCCCTGGA -3′
miR-199a-3p mimics	Sense	5′- ACAGTAGTCTGCACATTGGTTA -3′
	Antisense	5′- ACCAATGTGCAGACTACTGTTT -3′

### Animals

The Model Animal Center of Nanjing University commercially provided the 5-week-old BALB/c-nu female nude mice, and these mice were then kept in a special environment free of pathogens for animals, in which the mice had free access to food and water. One mouse was injected subcutaneously with a total of Huh-7/DDP cells (1 × 10^7^). The prepared cell suspension was subcutaneously injected to axillary of nude mice. Fourteen days later, the nude mice were undergoing tail intravenous injection with 20 μg exosome (suspended in 40 μl PBS) or PBS every 2 days, and were intraperitoneally injected with 5 mg/kg DDP every 4 days. After exosome injection, the tumor size was measured every 2 days. After 28 days of injection, the animals were killed. The tumor was excised and cut into slices (diameter: 2 mm). Ultimately, the slices were embedded into the subcutaneous region in the back of mice selected for following assays. The mice were anesthetized with diethyl ether. Finally, the xenograft tumors were removed after the mice were killed by cervical dislocation. The above steps were operated by reference to the guideline with the approval of the Institutional Animal Care and Research Advisory Committee of Zhejiang Provincial People’s Hospital. Animal experiments took place in SPF Animal Laboratory at Zhejiang University School of Medicine.

RETRACTED

### Statistical processing

From at least three independent assays, data were gained and expressed as mean ± SE. Student’s *t* test was executed for data comparisons, and *P*<0.05 displayed that there was a statistically significant difference; *P<0.05, **P<0.01 and ***P<0.001.

## Results

### Expression levels of miR-199a-3p in different cells and its possible targets

Aberrant expression of miRNAs has relationship to multi-drug resistance in HCC [39], and miR-199a-3p represses various malignant tumors. Hence, miR-199a-3p level in HL-7702, Huh-7 and Huh-7/DDP was examined via qRT-PCR. It was unraveled that miR-199a-3p level was attenuated in Huh-7 and evidently down-regulated in Huh-7/DDP relative to HL-7702 (Figure 1A), implying that miR-199a-3p may participate in the mechanism of HCC and DDP resistance. In order to examine the possible target genes of miR-199a-3p, several target genes of miRNAs were obtained by retrieving in the bioinformatics software Targetscan, PicTar, PITA, microT and miRmap, and related graphs were plotted (Figure 1B). Literature has revealed that ZEB1 [40], MTOR [41] and DNMT3A [42] are closely related to drug resistance of tumors. Subsequently, WB was implemented to ascertain these possible targets in Huh-7 and Huh-7/DDP cells. The results suggested that the expression of ZEB1, MTOR and DNMT3A was significantly higher in Huh-7/DDP cells than that of Huh-7 cell treated with whether in NC or miR-199a-3p mimics (Figure 1C–F).

**Figure 1:** Expression of miR-199a-3p and its possible targets (**A**) Expression levels of miR-199a-3p in HL-7702, Huh-7 and Huh-7/DDP are tested via qRT-PCR. (**B**) Possible miR-199a-3p targets are predicted via bioinformatics analysis. (**C**) WB is executed to ascertain the underlying targets in Huh-7 and Huh-7/DDP cells. (**D–F**) WB gray analysis. (**G–I**) CCK-8 is adopted for the determination of HL-7702 (G), Huh-7 (H) and Huh-7/DDP (I) cell viability under different drug concentrations, followed by calculation of inhibition rate; *P<0.05; **P<0.01; ***P<0.001. All error bars are s.e.m.

RETRACTED

### MiR-199a-3p mimics made HCC cells sensitive to DDP

Huh-7 and Huh-7/DDP cells in the 96-well plate were treated with miR-199a-3p mimics and NC mimics to work out the function role of miR-199a-3p. One day later, considering initial assay results, each plate well was added with DDP at different concentrations. Dual-dilution was executed to determine the range for HL7702, Huh-7 and Huh-7/DDP cells (0–12 μg/ml). After incubation for further 2 days, CCK-8 was implemented to examine cell viability, followed by calculation of inhibition ratio. Cell viability was attenuated in a concentration-dependent manner. The results revealed that cell viability was significantly inhibited by miR-199a-3p mimics when compared with cells treated with miR-NC. However, because of the higher expression of miR-199a-3p in HL-7702 cells, the cells were more sensitive to DDP treatment whether in group NC or group miR-199a-3p mimics than Huh-7 and Huh-7/DDP (Figure 1G–I). To sum up, miR-199a-3p mimics is capable of making cell lines sensitive to DDP and predominantly overturning Huh-7/DDP cell drug resistance

### Exosome-delivered miR-199a-3p mimics conjugated cells and modulated possible targets

After extracted from HEK293T cell medium, exosomes, which is a safer manner to transfer miR-199a-3p than chemical reagents, were identified by transmission electron microscopy(Figure 2A). WB results validated that relative to those in donor cells, the expressions of exosome labelled proteins were evidently elevated (Figure 2B). Besides, Huh-7 and Huh-7/DDP cell culture medium was added with PKH67-dyed exosomes, which conjugated the recipient cell cytoplasm and spread to numerous small stains on one side or surrounding the cell nucleus (Figure 2C). For miR-199a-3p transfer, HEK293T cells received treatment with NC mimics and miR-199a-3p mimics, and 2 days later, the secreted exosomes were obtained. Next, it was ascertained by qRT-PCR that miR-199a-3p expression level was evidently up-regulated in exosomes originated from the medium of cells treated with miR-199a-3p mimics relative to cells treated with NC mimics (Figure 2D). Finally, identical to the regulation by direct treatment with miR-199a-3p mimics, exosome-delivered miR-199a-3p mimics (exo-199a-3p mimics) were also able to down-regulate possible target protein expressions (Figure 2E,F).

**Figure 2:** Exo-miR-199a-3p mimics fuse into cells and modulate possible targets (**A**) Images of HEK293T cell medium exosomes under a transmission electron microscope. (**B**) Labeled proteins for exosomes are determined via WB and assessed by gray analysis. (**C**) Exosomes stained with PKH67 fused into HCC cells. (**D**) Measurement of miR-199a-3p expression levels in HEK exosomes by qRT-PCR. (**E** and **F**) Possible target protein expression levels in Huh-7 (E) and Huh-7/DDP (F) cells are tested by WB; **P<0.01; ***P<0.001. All error bars are S.E.M.

RETRACTED

### Exo-199a-3p mimics overturned the resistance of HCC cells to DDP

In light of the findings of CCK-8 assay (Figure 1G,H), when concentration was 3 μg/ml, the difference between the NC-mimics and miR-199a-3p-mimics groups was the most obvious, particularly for Huh-7/DDP cell transfection, so 3 μg/ml was considered to be the appropriate DDP concentration for subsequent application. First, the implemented CCK-8 assay validated that cell viability became predominantly weakened reduced by exo-199a-3p mimics in Huh-7 (Figure 3A) and Huh-7/DDP cells (Figure 3B). Besides, Huh-7/DDP cell viability was evidently higher than Huh-7 cell viability, and this finding was continuously demonstrated by 5-ethynyl-2′-deoxyuridine (EdU) assay (Figure 3C,D). Afterwards, Transwell assay was adopted for examining cell ability to invade, the results of which unraveled that the invasion capacity of Huh-7 cells undergoing co-incubation with DDP (3 μg/ml) and exosomes (exo-mock) untreated or those treated with miR-199a-3p/NC mimics became weakened. Moreover, in two control groups, Huh-7/DDP cells had strong capacity to invade, but exo-199a-3p mimics pronouncedly caused the drug sensitivity and magnifying the invasion repression of DDP (Figure 3E,F). Furthermore, the Huh-7 cell apoptosis rate was extremely high, and the apoptotic cell ratio slightly increased with exo-199a-3p mimics (Figure 4A,C). Additionally, exo-199a-3p mimics overturned DDP resistance and obviously increased the apoptotic Huh-7/DDP cells (Figure 4B,D).

**Figure 3:** Exo-199a-3p mimics overturn the resistance to DDP in HCC cells (**A**) Huh-7 cell viability detected by CCK-8 experiment. (**B**) Huh-7/DDP cell viability. (**C** and **D**) Cell proliferation is examined via EdU assay in Huh-7 and Huh-7/DDP cells. (**E** and **F**) Examination of the two cell lines invasion capacity via Transwell assay; **P<0.01, ***P<0.001. All error bars are S.E.M.

**Figure 4:** Exo-199a-3p mimics enhance the cytotoxicity of DDP in HCC cells (**A** and **B**) Cell apoptosis is tested through TUNEL in Huh-7 and Huh-7/DDP cells. (**C** and **D**) Quantitative assessment of cell apoptosis; **P<0.01; ***P<0.001. All error bars are S.E.M.

### Systemically injected exo-199a-3p triggered the sensitivity to DDP *in vivo*

*In vivo*, Huh-7/DDP were injected to construct nude mouse models of tumor (*n*=3, each group) followed the steps of Figure 5A. In accordance with the formula, the tumor volume was calculated, and every other day the tumor major and minor axes were recorded. As time passed, it was discovered that control group had progressive tumors while treatment group had stable tumors (Figure 5B). Thereafter, each group of tumors and blood were harvested for later tests, followed by tumor photographing (Figure 5C), and the systemic injection of exo-199a-3p mimics resulted in markedly minor tumors (Figure 5D). What’s more, the systemically injected exo-199a-3p mimics led to significantly less lung metastasis nodes (Figure 5E). Subsequent to extraction of exosomes from mouse serum, the high level of miR-199a-3p (Figure 5F) in exosomes from the exo-199a-3p mimics group was validated through qRT-PCR. Consequently, miR-199a-3p expression level in tumors was pronouncedly upregulated (Figure 5G), and its possible target proteins were down-regulated in treatment group (Figure 5H), functioning as a possible mechanism by which sensitivity to DDP was enhanced in the body.

RETRACTED

**Figure 5:** Systemically injected exo-199a-3p mimics cause sensitivity to DDP (**A**) A flow chart depicting the *in vivo* experimental design. (**B**) Changes in the tumor volume in control and treatment groups. (**C**) Mouse tumor images (*n*=3, each group). (**D**) Tumor weight measurement. (**E**) Lung metastasis nodes. (**F**) Levels of miR-199a-3p in serum exosomes are assessed by qRT-PCR. (**G**) MiR-199a-3p expression level in tumors. (**H**) Immunohistochemistry analysis of possible target proteins; *P<0.05; **P<0.01; ***P<0.001. All error bars are s.e.m.

## Discussion

Primarily because of chemoresistance (like DDP resistance), the death rate of HCC remains high [43]. The resistance mechanism in cells triggered by many factors such as the abnormally expression miRNAs [20]. Besides, compared with HL-7702 cells, miR-199a-3p expression level was found to gradually decrease in the Huh-7 and Huh-7/DDP cells, revealing an underlying mechanism in the therapy resistance to DDP. Hence, up-regulation of miR-199a-3p is likely to be a new way for the improvement of the sensitivity to chemotherapy. Direct treatment of HCC cells with miR-199a-3p mimics could elevate the inhibition rate resulted from DDP. After extraction of exo-199a-3p mimics, a train of assays denoted that these mimics were able to weaken the cell viability and slowed down invasion, but facilitated apoptosis in the body. Additionally, mice were injected with exo-199a-3p mimics through the tail vein and intraperitoneally injected with DDP, which overturned the chemoresistance in the body. Further, screening for possible target genes of miR-199a-3p in HCC cells were conducted via bioinformatics analysis. Through the literature review, three of them were reported to be involved in the chemoresistance. Previous research pointed out ZEB1 confers chemotherapeutic resistance to breast cancer by activating ATM [40]. Similar mTOR [41,44] and DNMT3A [42,45] have also been shown to promote tumor resistance. Subsequently, WB and other experiments confirmed that miR-199a-3p mimics and exo-199a-3p mimics could reduce their expressions. It can be concluded from the present study that miR-199a-3p may inhibit tumor resistance by silencing ATM, mTOR and DNMT3A expressions.

RETRACTED

The possible application of miRNAs in drug-refractory cancer has been brought into focus. MiR-488 represses HCC cells to proliferate and generate DDP sensibility by activating the NER signaling pathway mediated by eIF3a [46]. Decrement of miR-196a strengthens the sensitivity of HCC cells to DDP treatment [47]. Viral vectors [48] and liposomal carriers [49] have been widely applied to transfer certain miRNAs and adjust the expression of them, but unfavorable biocompatibility, non-exact cytotoxicity and low transferring efficacy remain difficult to overcome for delivering miRNAs in the body [50]. In the present research, mice received intravenous injection of exosomes separated from cell culture medium, thus raising miR-199a-3p expression in tumors and exosomes, which may be a less cytotoxic treatment regimen with better biocompatibility. As such, exo-199a-3p mimics remained stable in the blood and caused an elevation of miR-199a-3p expression in mice tumors, triggering the sensitivity of refractory tumors to DDP. Ultimately, cell invasion, apoptosis and viability were tested to work out the probable mechanisms by which HCC is resistant to DDP. Results showed that miR-199a-3p promoted apoptosis and inhibited cell viability and invasion. The most possible explanation or the interaction of different mechanisms needs to be investigated in the future.

In conclusion, exosome-delivered miR-199a-3p mimics overturn the HCC resistance to DDP, speed up cell apoptosis and slow down invasion outside the body and tumor growth in the body, which is considered to be an underlying method in DDP-resistant HCC therapy in the future.

## Data Availability

The data in the current study are available from the corresponding authors on reasonable request.

## Abbreviations

CCK-8: Cell Counting Kit-8
EdU: 5-ethynyl-2′-deoxyuridine
HCC: hepatocellular carcinoma
miRNA: micro RNA
ncRNA: non-coding RNA
WB: Western blotting
